# Characterization of lncRNA-Based ceRNA Network and Potential Prognostic Hub Genes for Sepsis

**DOI:** 10.1155/2022/1485033

**Published:** 2022-06-21

**Authors:** Yiqing Tong, Yanping Yang, Qiming Feng

**Affiliations:** Emergency Department, Shanghai Jiaotong University Affiliated Sixth People's Hospital, Shanghai, China

## Abstract

**Objective:**

Sepsis is one of the most common reasons for hospitalization and in-hospital mortality each year. Noncoding RNAs have been reported not only as diagnostic and prognostic indicators but also as therapeutic targets of sepsis. Herein, we used an integrative computational approach to identify miRNA-mediated ceRNA crosstalk between lncRNAs and genes in sepsis based on the “ceRNA hypothesis” and investigated prognostic roles of hub genes in sepsis.

**Methods:**

Two good-quality gene expression datasets with more than 10 patient samples, GSE89376 and GSE95233, were employed to obtain differentially expressed lncRNAs (DElncRNAs) and genes (DEGs) in sepsis. The DElncRNA-miRNA-DEG regulatory network was constructed using a combination of DElncRNA-miRNA pairs and miRNA-DEmRNA pairs. The protein-protein interaction (PPI) network was constructed by mapping DEGs into the STRING database to identify hub genes in sepsis. The clinical and prognostic significance of hub genes was validated in 89 patients with post-traumatic sepsis.

**Results:**

The integrative computational approach identified 311 DEGs and 19 DElncRNAs between septic patients and healthy volunteers. Results yielded 122 downDElncRNA-miRNA-downDEG networks based on two lncRNAs, HCP5, and HOTAIRM1, and 36 upDElncRNA-miRNA-upDEG network based on BASP1-AS1. The PPI network identified serum/glucocorticoid regulated kinase 1 (SGK1), arrestin beta 1 (ARRB1), and G protein-coupled receptor 183 (GPR183) as located at the core of the network, and three of them were downregulated in sepsis. SGK1, ARRB1, and GPR183 were all involved in lncRNA HCP5-based ceRNA network. The quantitative real-time PCR revealed that the patients with post-traumatic sepsis exhibited reduced relative mRNA levels of SGK1, ARRB1, and GPR183 compared to the patients without sepsis. The nonsurvivor group, according to the 28-day mortality, showed lower relative mRNA levels of SGK1, ARRB1, and GPR183 than the survivor group. We also demonstrated reduced mRNA levels of SGK1, ARRB1, and GPR183 were associated with sepsis-related death after trauma.

**Conclusion:**

Our integrative analysis and clinical validation suggest lncRNA HCP5-based ceRNA networks with SGK1, ARRB1, and GPR183 involved were associated with the occurrence and progression of sepsis.

## 1. Introduction

Initially, sepsis was thought to be an infectious process of systemic inflammatory response syndrome. This definition was agreed upon in an ACCP/SCCM (American College of Chest Physicians/Society of Critical Care Medicine) Consensus Conference in 1991 [1]. At the Third International Conference in 2016, sepsis was defined as the life-threatening organ dysfunction caused by the host's maladjusted response to infection and it was mainly characterized by organ failure in clinical [2]. Sepsis easily transits into septic shock if without timely treatment. Septic shock is defined as a subset of sepsis and the severest condition of sepsis, which results in 40% or more deaths [3]. The specific populations such as infants [4] and elders [5] are prone to be attacked by sepsis might be due to compromised immune systems. Furthermore, increasing studies reveal there is a gender specific difference in the incidence rate of infectious diseases [6, 7]. Females run a lower risk of developing most infectious diseases including sepsis than males, which is mainly associated with hormones. Androgen has been shown to inhibit cell-mediated immune responses while estrogen has a protective effect on immune cells [8].

Sepsis is a global medical problem and remains the leading cause of death induced by infection. Early recognition and diagnosis of sepsis are still the main approaches to reduce mortality. Molecular detection can not only be used as an effective method for early diagnosis and preliminary evaluation of sepsis but also as a tool to judge whether there is potential infection in inflammatory patients by analyzing biomarkers. Epigenetic regulation of long noncoding RNA (lncRNA) has been proven in a variety of immune-related diseases. For example, lncRNA E330013P06 promoted proinflammatory in type 2 diabetic mice by regulating expression of inflammation related gene [9]. Circulating lncRNA ZFAS1 knockdown was associated with increased inflammatory response and worse prognosis in sepsis patients. Furthermore, ZFAS1 also presented a good diagnostic value for sepsis [10]. As a vital immunomodulatory factor, lncRNA NEAT1 was found to be unregulated in septic patient. It can be used as a biomarker to distinguish sepsis patients from patients with systemic inflammatory response syndrome [11]. In recent years, competing endogenous RNAs (ceRNAs) have aroused huge concern in medical science. CeRNA network is beneficial for detection of biomarkers in various diseases [12, 13]. This study attempts to deeply understand the molecular regulatory network in the infection process of sepsis, and hence we perform integrative computational approach to identify the lncRNA-based ceRNA network in sepsis.

## 2. Materials and Methods

### 2.1. Data Source, Data Processing, and Differential Analysis

The gene expression datasets used in this study were downloaded from the Gene Expression Omnibus (GEO) database. Firstly, we used the term “sepsis” as a keyword to search GEO Accession and selected “Homo sapiens” as the specimen. Next, we selected datasets GSE89376 and GSE95233 both of which have more than 10 patient samples. The GSE89376 contains gene expression profile data derived from sepsis and normal control (*n* = 12 for each), which was generated in the GPL22628 platform. GSE95233 was generated in the GPL570 platform and assembled gene expression profile data from 51 cases of septic shock and 22 normal controls. The raw data of two datasets were handled, normalized, and log2-transformed. The Limma package of the R/Bioconductor software was conducted to analyze differentially expressed lncRNAs (DElncRNAs) and genes (DEGs). The genes with |log2 (fold change (FC)| > 1.5 and corrected *P* < 0.05 were regarded as initial DElncRNAs or DEGs.

### 2.2. Construction of the circRNA-miRNA-mRNA ceRNA Network

Putative DElncRNA-miRNA pairs were predicted by mapping DElncRNAs into the Starbase database. Putative miRNA-DEmRNA pairs were predicted by mapping DEmRNA into the miRMap, miRanda, miRDB, TargetScan, and miTarBase, and overlapping pairs were regarded as final miRNA-DEmRNA pairs. The DElncRNA-miRNA-DEG regulatory network was constructed using a combination of DElncRNA-miRNA pairs and miRNA-DEmRNA pairs according to the principle of the ceRNA network and visualized using the cytoscape3.4.0 software.

### 2.3. Functional Annotation

Gene ontology (GO) and Kyoto Encyclopedia of Genes and Genomes (KEGG) enrichment analyses were carried out to integrate significant genes with a specific function through the database for annotation, visualization, and comprehensive discovery (DAVID).

### 2.4. Protein-Protein Interaction (PPI) Network Construction

The search tool for the retrieval of interacting genes (STRING online tool) is used to annotate the functional interactions between predictive proteins and known proteins, and then the PPI network analysis was performed to reflect significant interactions of hub genes.

### 2.5. Study Subjects

The clinical study included 189 patients with multiple traumas who were admitted into the EICU of Shanghai Sixth People's Hospital from January 2020 to September 2021, with the approval of the Ethics Committee. Each patient among 189 patients, 89 developed post-traumatic sepsis. The diagnosis of sepsis was made as previously reported [2]. The SOFA scores that reflect the function of an organ system and range from 0 to 4 are obtained on admission to ICU and at a period of 24 h. These 89 patients with sepsis were followed up to record the 28-day mortality. Informed consent was obtained from patients or their legal guardians.

### 2.6. Blood Sample Collection and Quantitative Real-Time PCR

The patient serum was added with Trizol reagents (Thermo Fisher Scientific, USA) to isolate total RNA. Using the PrimeScript RT Reagent kit (Takara, Dalian, China), the cDNA was generated. Then, qPCR was carried out using the SYBR® Premix Ex Taq™ II kit (Takara) and a ABI PRISM®7500 System (Applied Biosystems, Foster City, CA, USA). The primer sequences (SGK1: sense, 5′-GCCAAGTCCCTCTCAACAAATCA-3′ and antisense, 5′-GTGCCTAGCCAGAAGAAGAACCTTT-3′; ARRB1: sense, 5′-GCGAGCACGCTTACCCTTT-3′ and antisense, 5′-CAAGCCTTCCCCGTGTCTTC-3′; GPR183: sense, 5′-GAAGAAGACGACGACCGCAA-3′ and antisense, 5′-GGATCCATGGAGTACTTGCAGA-3′; *β*-actin: forward, 5′-GTCTTCCCCTCCATCGTG-3′ and reverse, 5′-AGGGTGAGGATGCCTCTCTT-3′) were obtained from Invitrogen (USA). Relative mRNA expressions of SGK1 and ARRB1 to the house-keeping gene *β*-actin were determined by the 2^−ΔΔCt^ methods.

### 2.7. Statistical Analysis

A manner of the mean ± standard deviation (for measurement data) or ratio (for enumeration data) was used to present the data. The measurement data was analyzed by the *t*-test and the enumeration data by the chi-square test. The Kaplan–Meier method followed by a log-rank test was used to estimate the 28-day mortality of sepsis patients according to the mRNA levels of SGK1, ARRB1, and GPR183. Statistical analysis was performed using the SPSS 19.0 software package (IBM, USA) and figure creation was performed using GraphPad Prism Version 8. A possibility (*P*) < 0.05 reflects a significant difference.

## 3. Results

### 3.1. Identification of DEGs and DElncRNAs in Sepsis

After differentially analyzing the raw data deposited in the GSE89376 and GSE95233 datasets, initial DEGs fulfilling |log^2^(FC)| > 1.5 and corrected *P* < 0.05 between septic patients and healthy volunteers were presented by volcano plots (Figure 1(a)) and their expression diversity was shown by heatmaps (Figure 1(b)). Overlapping DEGs, including 119 downregulated DEGs and 192 upregulated DEGs, between GSE89376 and GSE95233 datasets were considered as final DEGs between septic patients and healthy volunteers (Figure 1(c)). We continued to differentially analyze the GSE89376 and identify 19 DElncRNAs (14 downregulated DElncRNAs and 5 upregulated DElncRNAs) fulfilling |log2(FC)| > 1.5 and corrected *P* < 0.05 between septic patients and healthy volunteers (Figures 2(a) and 2(b)).

### 3.2. Construction of DElncRNA-miRNA-DEG Regulatory Network in Sepsis

To investigate the ceRNA network in the context of sepsis, we first mapped 311 DEGs between septic patients and healthy volunteers into miRMap, miRanda, miRDB, TargetScan, and miTarBase databases and identified 2064 overlapping pairs of interacting miRNAs and DEGs (690 pairs based on downregulated DEGs and 1374 pairs based on upregulated DEGs) in at least four databases concurrently. We next mapped 19 DElncRNAs into the Starbase database and identified 97 pairs of interacting DElncRNAs and miRNAs (89 pairs based on downregulated DElncRNAs and 8 pairs based on upregulated DElncRNAs). As the ceRNA hypothesis showed, lncRNAs sponge miRNA and affect post-transcriptional control. There are two paradigms of regulation: the downlncRNA-miRNA-downgene network and the uplncRNA-miRNA-upgene network. Therefore, we intersected 2064 miRNA-DEG interactions and 97 lncRNA-mRNA interactions to construct the DElncRNA-miRNA-DEG network in sepsis. Results yielded 122 downDElncRNA-miRNA-downDEG networks based on two lncRNAs, HCP5 and HOTAIRM1, (Figure 3(a)), and 36 upDElncRNA-miRNA-upDEG networks based on BASP1-AS1 (Figure 3(b)).

### 3.3. Enrichment Analysis in Sepsis

We performed GO annotation and KEGG pathway analyses to assess the main functional pathways of DEGs involved in the ceRNA network related to sepsis. GO analysis revealed that the DEGs between septic patients and healthy volunteers were enriched in 200 GO terms (*P* < 0.05), including 172 terms belonging to BP, 8 terms to CC, and 20 terms to MF.  Figure 4(a) lists top 15 GO terms which were enriched by DEGs, such as secretory granule localization, positive regulation of ERK1 and ERK2 cascade, oxysterol binding, and purine ribonucleotide binding.  Figure 4(b) lists top 15 KEGG pathways which were enriched by DEGs (*P* < 0.05) including MAPK signaling pathway, morphine addiction, and parathyroid hormone synthesis secretion and action.

### 3.4. PPI Network

As shown in the PPI network, 3 hub genes located at the core of the network with three interactions were identified, including serum/glucocorticoid regulated kinase 1 (SGK1), arrestin beta 1 (ARRB1), and G protein-coupled receptor 183 (GPR183) (Figure 5), and three of them were downregulated in sepsis. SGK1, ARRB1, and GPR183 were all involved in lncRNA HCP5-based ceRNA networks, including HCP5-miR-29a/b/c-3p-SGK1, HCP5-miR-323a-3p/miR-520a-5p/miR-525-5p-SGK1, and HCP5-miR-144-3p-GPR183.

### 3.5. The Expression Levels of Hub Genes in Septic Patients

No significant difference in age, gender distribution, BMI, cause and location of trauma between traumatic patients with or without the incidence of sepsis was noted (*P* > 0.05). The quantitative real-time PCR was performed to determine the mRNA levels of SGK1, ARRB1, and GPR183 in the serum of patients with or without post-traumatic sepsis. The relative mRNA levels of SGK1, ARRB1, and GPR183 in patients with post-traumatic sepsis were 3.88 ± 0.47, 2.76 ± 0.32, and 2.17 ± 0.24. The relative mRNA levels of SGK1, ARRB1, and GPR183 in traumatic patients without sepsis were 5.85 ± 0.30, 3.98 ± 0.45, and 3.42 ± 0.31, respectively. It was revealed that the patients with post-traumatic sepsis exhibited reduced relative mRNA levels of SGK1, ARRB1, and GPR183 compared to the patients without sepsis (Figure 6(a), *P* < 0.001).

### 3.6. Prognostic Performance of Hub Genes for Sepsis

We classified 89 sepsis patients into survivor and nonsurvivor groups based on the 28-day mortality. The two groups exhibited no significant difference in demographic data (*P* > 0.05). The relative mRNA levels of SGK1, ARRB1, and GPR183 in the survivor group were 4.00 ± 0.44, 2.82 ± 0.31, and 2.22 ± 0.25, respectively. The relative mRNA levels of SGK1, ARRB1, and GPR183 in the nonsurvivor group were 3.62 ± 0.41, 2.62 ± 0.30, and 2.07 ± 0.20, respectively. As shown in Figure 6(b), the nonsurvivor group showed lower relative mRNA levels of SGK1, ARRB1, and GPR183 than the survivor group (*P* < 0.05). The cumulative risk of 28-day mortality for patients with post-traumatic sepsis according to the relative mRNA levels of SGK1 (with 3.87 as a cutoff), ARRB1 (with 2.76 as a cutoff), and GPR18 (with 2.17 as a cutoff) was estimated. It was noted that reduced mRNA levels of SGK1, ARRB1, and GPR183 were associated with sepsis-related death after traumas (Figure 7, (*P* < 0.05).

## 4. Discussion

Sepsis is a serious infection response with high morbidity and mortality. Rapid diagnosis and urgent intervention are very important to improve the prognosis [14]. Although rapid and accurate analysis of pathogens causing infection remains a major challenge in modern health care, molecular detection has created a new progress in diagnosis of sepsis by improving early intervention performance and reducing mortality [15, 16].

Recent studies indicate that lncRNAs were involved in the process of sepsis infection through regulating expression of proinflammatory genes [17, 18]. Increasing studies demonstrated circulating microRNAs (miRNAs) could be used as potential biomarkers of sepsis [19, 20]. It was found that close interaction exists between mRNAs and noncoding RNAs represented by lncRNAs, miRNAs, and circular RNAs (circRNAs). These molecules regulate each other's expression by competing microRNAs (miRNAs) and the process is defined as ceRNA hypothesis [21]. This study tried to investigate the role of ceRNA regulator network in sepsis, thereby, according to ceRNA hypothesis, the present study constructed a DElncRNA-miRNA-DEG regulatory network through an integrative computational approach, and identified hub genes based on PPI network in sepsis. The data showed three downregulated genes including SGK1, ARRB1, and GPR183 were involved in lncRNA HCP5-based ceRNA networks consisting of HCP5-miR-29a/b/c-3p-SGK1, HCP5-miR-323a-3p/miR-520a-5p/miR-525-5p-SGK1, and HCP5-miR-144-3p-GPR183. Protein kinase plays a major regulatory role in cell biology and it's one of the most important drug targets in the pharmaceutical industry. Protein kinases stimulate or inhibit their functions by phosphorylating other proteins, thus affecting many different biological processes [22]. SGK1 belongs to AGC protein kinase family and phosphorylates serine and threonine residues of targeted proteins. It is well known that it plays a regulatory role in numerous ion channels and transporters [23]. In a study of rat hippocampal neurons in vitro and in vivo, Zhang et al. [24] indicated SGK1 overexpression contributed to the decrease of apoptosis of neurons cells following glucose deprivation or ischemia reperfusion. Additionally, its role in inhibiting apoptosis was mediated by the PI3K/Akt/GSK3*β* pathway. Impact of SGK1 on insulin sensitivity has been identified and this study showed liver-specific SGK1-knockout mice had glucose intolerance and insulin resistance [25]. Sepsis is a fatal inflammatory reaction associated with immune dysfunction. Autophagy has been shown to be closely related to inflammation and immunity. Autophagy is involved in chronic human diseases, including infection, cancer, heart disease and neurodegeneration [26]. Elevated autophagy associated with reduced inflammatory response in patients with sepsis [27]. Recent studies showed SGK1 is a switch for stable autophagy [23]. The results of quantitative real-time PCR in our study found that the patients with post-traumatic sepsis showed decreased relative mRNA expression of SGK1 in serum. Our findings might demonstrate that reduced autophagy occurred in the sepsis patients. Previous study manifested that acute lung injury induced by sepsis was alleviated through activation of SIRT1/SGK1/Nedd4-2 signaling pathway [28]. Wang and Han also confirmed that upregulated SGK1 suppressed inflammation induced by doxorubicin [29]. In the present study, we observed relative mRNA levels of ARRB1 and GPR183 were downregulated in the patients with post-traumatic sepsis. Arrestin family includes arrestin−1 to −4, which is a scaffold protein originally found to play a role in G protein-coupled receptor desensitization. Arrestin-2, also known as arrestin beta 1 (ARRB1), plays a broader role in cell signaling [30]. It has recently been found to be involved in the pathogenesis of various inflammatory diseases. A study presented decreased levels of inflammatory cytokine in ARRB1 and arrestin beta 2 silence mice after administration of lipopolysaccharide [31]. The conclusion above was supported by another study. The absence of ARRB1 expression in nonhematopoietic cells leads to activation of inflammatory factors in mice, and induce more mortality of mice in polymicrobial sepsis model [32]. GPR183 (EBI2) is a seven transmembrane G protein-coupled receptor and mediates migration of immune cells [33]. Bartlett et al. pointed out the patients with tuberculosis and type 2 diabetes revealed reduced GPR183 levels. The mice with GPR183 deficiency are associated with increased *Mycobacterium tuberculosis* and immune dysregulation [34]. Enormous studies have confirmed GPR183 is a therapeutic target for inflammatory and metabolic diseases [35, 36]. The prognosis function of SGK1, ARRB1, and GPR183 was well established in various diseases such as prostate cancer, lung cancer, and breast cancer [37–39]. In our prognostic analysis, the nonsurvivor group revealed lower expression of SGK1, ARRB1, and GPR183 than the survivor group, and was at higher risk of sepsis-induced death.

There are two limitations needed to inform when interpreting our results. On the one hand, the sample size of clinical human blood for RT-qPCR validation of lncRNAs of interest was relatively small, which may weaken the reliability of clinical data. On the other hand, given the preliminary nature of our study, further functional studies were required to elucidate sepsis pathogenesis focusing on lncRNA-based ceRNA action.

In conclusion, lncRNA-based ceRNA network is beneficiary to deeply understand the molecular regulatory network in sepsis infection, and its hub genes including SGK1, ARRB1, and GPR183 contributed to distinguish sepsis group from nonsepsis group. These hub genes might be considered as potential biomarker for sepsis diagnosis and risk factors of sepsis death. Next, we will further elaborate the specific signal mechanism of these three genes in the process of sepsis infection.

## Figures and Tables

**Figure 1:** Identification of DEGs between sepsis and normal control by differentially analyzing the GSE89376 and GSE95233 datasets. (a) The volcano plots of DEGs; (b) the heatmaps showing expression diversity of DEGs. (c) Venn diagram showing overlapping DEGs including 119 downregulated DEGs and 192 upregulated DEGs between sepsis and normal control in two datasets.

**Figure 2:** Identification of DElncRNAs between sepsis and normal control by differentially analyzing the GSE89376. (a) The volcano plots of DElncRNAs; (b) the heatmaps showing expression diversity of DElncRNAs.

**Figure 3:** Construction of DElncRNA-miRNA-DEG regulatory network in sepsis, including 122 downDElncRNA-miRNA-downDEG networks (a) and 36 upDElncRNA-miRNA-upDEG networks (b).

**Figure 4:** The DEGs among the DElncRNA-miRNA-DEG regulatory network in sepsis were analyzed by GO annotation and KEGG pathway. (a) GO annotation. (b) KEGG pathway.

**Figure 5:** The PPI network of DEGs involved in the ceRNA network related to sepsis.

**Figure 6:** The quantitative real-time PCR was performed to determine the mRNA levels of SGK1, ARRB1, and GPR183 in the serum of patients with (*n* = 89) or without post-traumatic sepsis (*n* = 100) (a), in the serum of survivors (*n* = 29) or nonsurvivors (*n* = 60) during 28 days (b). ^*∗*^indicates *P* < 0.05.

**Figure 7:** The Kaplan–Meier curves plotting the 28-day mortality of sepsis patients based on the relative mRNA levels of SGK1 (with 3.87 as a cutoff), ARRB1 (with 2.76 as a cutoff), and GPR18 (with 2.17 as a cutoff).

## Data Availability

The data used to support the findings of this study are included within the article.
